# Comprehensive Analysis of Regulatory Network for LINC00472 in Clear Cell Renal Cell Carcinoma

**DOI:** 10.1155/2021/3533608

**Published:** 2021-06-09

**Authors:** Shuoze Gao, Zhiping Wang

**Affiliations:** Institute of Gansu Nephro-Urological Clinical Center, Department of Urology, Institute of Urology, Key Laboratory of Urological Disease of Gansu Province, Lanzhou University Second Hospital, Lanzhou, China

## Abstract

Renal cell carcinoma (RCC) accounts for about 2% to 3% of adult malignancies, and clear cell renal cell carcinoma (ccRCC) is the most common and aggressive type of kidney cancer. It accounts for 75% of all kidney tumors. Although new targeted drugs continue to appear, they are still not suitable for all patients. Therefore, an in-depth study of the molecular mechanism of the development of ccRCC and exploration of new targets for the treatment of ccRCC will help to achieve precise treatment for ccRCC. With the development of molecular research, the study of long noncoding RNA (LncRNA) has given us a new understanding of tumors. Although LncRNA does not encode proteins, it directly interacts with proteins in various signaling pathways and affects cell functions. Therefore, it is of great significance to study the mechanism of LncRNA in ccRCC. The expression level of Linc00472 in ccRCC tissues is significantly lower than adjacent normal tissues, and its low expression is closely related to Furman's high grade. The low expression of Linc00472 is associated with poor prognosis in patients with ccRCC. The results of protein interaction and functional enrichment analysis indicate that genes upregulated in renal clear cell carcinoma may play a major role. Analysis of target gene prediction results showed that Linc00472 may be used as ceRNA in the miR-24-3p-HLA-DPB1 pathway, miR-24-3p-CXCL9 pathway, miR-221-3p-C3aR1-VEGFR2 pathway, miR-17-5p-HLA-DQA1/HLA-DQB1 pathway, and miR-17-5p-C3aR1/C5aR1-VEGFR2 pathway which play important functions. In addition, the regulatory relationship between miR-24-3p and TNFR2 (TNFRSF1B), CD36, and COL4A1 should also be noted. The value of Linc00472 in the diagnosis and treatment of ccRCC is worthy of further study.

## 1. Introduction

Renal cell carcinoma (RCC) accounts for about 2% to 3% of adult malignant tumors, and clear cell renal cell carcinoma (ccRCC) is the most common and aggressive type of renal carcinoma. It accounts for 75% of all kidney tumors [1, 2]. In recent years, the incidence of renal cancer has been on the rise in China, which presents higher requirements for its prevention and treatment. With the development of molecular research, modern oncology is being further improved, and these studies may have a profound impact on the prevention and treatment of tumors. Especially, the research on long noncoding RNA (LncRNA) is improving our understanding of kidney cancer. However, there are still many factors that hinder the realization of this goal. In particular, the regulatory mechanism of gene expression is still unknown; it is a major challenge to construct a multi-molecule regulatory network, and targeted therapy is not always effective for patients.

As an RNA transcript that is not translated into protein, LncRNA is more specific than messenger RNA (mRNA) in defining cell ontogeny and most protein-coding genes [3–5]. LncRNA affects cell functions through genome-wide transcriptional regulation and direct interaction with proteins in a variety of signaling pathways. In addition, the dysregulation of LncRNA expression in kidney cancer often leads to the promotion of a variety of carcinogenic mechanisms and the development of treatment resistance. Therefore, it is very important to understand the role of LncRNA in kidney cancer, which will help strengthen the prevention and treatment of kidney cancer.

Compared with the highly expressed LncRNA in kidney cancer, the research on the low expression of LncRNA is still less and not in-depth. Therefore, we focused on studying the low expression of LncRNA in renal clear cells, and found LncRNA-Linc00472, which is worthy of further study. Through the analysis of data from multiple public databases and the detection of the expression level of Linc00472 in ccRCC on collected tissue specimens, we have initially constructed the regulatory network of Linc00472 in renal clear cell carcinoma for further study of Linc00472 in ccRCC. The mechanism of action in cell carcinoma and its influence on the diagnosis, treatment, and prognosis of ccRCC provide a theoretical basis in bioinformatics [6].

## 2. Materials and Methods

### 2.1. Data Source and Screening of DEGs

The TCGA (The Cancer Genome Atlas) database is a joint project initiated by the National Cancer Institute and the Human Genome Institute. TCGA sequenced the whole genome of a variety of tumors and made the sequencing results public for research around the world. The CRN (Cancer RNA-Seq Nexus) database is a comprehensive database jointly developed by the University of Southern California and National Chung Hsing University. CRN systematically collects genome sequencing results from TCGA, SRA (Solicitors Regulation Authority), and GEO (Gene Expression Omnibus) databases, and can directly analyze the expression profiles of tumor transcriptomes (including LncRNA) [7, 8].

Download LncRNA and protein- coding genes differentially expressed in ccRCC through the CRN database. The data comes from the RNA-seq expression profile of renal clear cell carcinoma (KIRC) in the TCGA database, including Furman grade I to IV, with a total of 529 cases of cancer tissues (265 cases of grade I, 57 cases of grade II, 126 cases of grade III, and 81 cases of grade IV) and 72 adjacent tissues. For the screening of LncRNA, ∣log2 (Fold Change)∣ ≥ 1, FPKM > 0.1, adjusted *P* < 0.01 is the standard; for the screening of protein-coding genes, ∣log2 (Fold Change)∣ ≥ 1, FPKM > 5, adjusted *P* < 0.01 is the standard. The finally obtained LncRNA and protein-coding genes need to be expressed in grades I to IV that meet the screening conditions.

### 2.2. The Expression and Correlation Analysis of Linc00472 in ccRCC

The GEPIA2 (Gene Expression Profiling Interactive Analysis 2) platform was developed by Peking University. It can directly analyze the RNA sequencing expression data of 9736 tumors and 8587 normal samples from the TCGA and GTEx (Genotype-Tissue Expression) databases [9].

The expression level of Linc00472 in 31 tumors was obtained through GEPIA2, and the data were derived from the RNA-seq expression profile of the TCGA database. The expression level of Linc00472 in tumor tissues and adjacent normal tissues was further obtained, and the expression difference of Linc00472 was analyzed in grades I to IV. Then, the survival analysis was performed on the high-expression group and the low expression group of Linc00472.

### 2.3. Collection of Organization and Clinical Data

In this study, a total of 22 cases of ccRCC tissues and paired adjacent tissues were collected from postoperative patients who had undergone surgery at the Second Hospital of Lanzhou University. The diagnosis and grading of all renal clear cell carcinoma tissues are confirmed by histopathology. Histopathological grading follows the Furman grading method.

After the renal clear cell carcinoma tissue specimens were taken out by the surgeon, tumor information was collected within 15 minutes. One part was used for pathological examination and the other part was placed in a cryotube and quickly transferred to a −80°C refrigerator for long-term storage. After obtaining the pathological results, the patient's basic information (including age, gender, tumor size, and pathological grade) is derived from the information management system of the Second Hospital of Lanzhou University to obtain the patient's complete clinical data.

### 2.4. Quantitative Real-Time Polymerase Chain Reaction

Total RNAs were extracted from clinical tissue samples and cell lines using TRIzol reagent (Takara, Dalian, China) and were reverse-transcribed into cDNA with a random primer and reverse transcriptase kit (Accurate, Hunan, China) according to the manufacturer's instructions. Then, quantitative real-time PCR was performed using TB Green Premix Ex Taq II (Accurate) at an Applied Biosystems 7500 Real Time PCR system based on the manufacturer protocols. The specific primers for LINC00472 were (forward) 5′- TTTTATCCTAGATTGCCACCAC -3′ and (reverse) 5′-TTAGCATCTAGGCCCAGGTT -3′. The specific primers for *β*-actin were (forward) 5′-CCCTGGACTTCGAGCAAGAGAT-3′ and (reverse) 5′-GTTTTCTGCGCAAGTTAGG -3′. Relative LINC00472 expression was normalized to *β*-actin.

### 2.5. Gene Ontology and Pathway Enrichment Analysis

The Co-LncRNA database collected RNA-seq data from 28 human tissues and a total of 29,012 samples, including 133 data sets from TCGA and 108 datasets from GEO. Predict the target gene of LncRNA by coexpression analysis, and analyze the biological function of LncRNA by enriching the target gene [10]. DAVID is an online gene annotation and function enrichment website developed by the LHRI team of Leidos Biomedical Research Company in the United States [11, 12]. Gene Ontology (Gene Ontology, GO) is a database established by the Gene Ontology Consortium, which can analyze the biological process (BP), molecular function (MF), and cytological components of genes (cellular components, CC) and carry out functional annotations [13]. Kyoto Encyclopedia of Genes and Genomes (KEGG) is a database established by the Bioinformatics Center of Kyoto University, Japan, which uses genetic information to make calculations and speculations on higher-level and more complex cell activities and biological behaviors. Among them, the KEGG Pathway database stores information on gene pathways in various species [14].

Download data on the coexpression relationship between LncRNA and mRNA identified by Spearman correlation analysis and linear regression correlation analysis through the Co-LncRNA database, and then screen out coexpressed mRNAs that are differentially expressed in grades I to IV (*P* < 0.01). The selected differential genes were analyzed by GO BP and KEGG Pathway enrichment analysis by DAVID, and the function and approach of *P* < 0.01 after correction by false discovery rate (FDR) were used to annotate the function of Linc00472 [15].

### 2.6. PPI Network Construction and Module Analysis

The STRING database is a database that analyzes protein-protein interaction (PPI). It collects, scores, and integrates all publicly available protein-protein interaction information, and supplements this information through computational predictions. Currently, the STRING database covers 24,584,628 proteins from 5,090 organisms [16, 17].

The coexpressed mRNAs that were differentially expressed in grades I to IV were correlated through the STRING database, and a visual PPI network was constructed by Cytoscope3.8 software. In addition, the analysis of the functional modules of the PPI network was performed through the MCODE application in the Cytoscope3.8 software. The MCODE setting parameters are as follows: degree of interaction cutoff = 2, node score cutoff = 0.2, the maximum depth (max depth) = 100, and the *k* value (*k*-score) = 2. Then, perform GO BP and KEGG Pathway enrichment analysis on the differential proteins in the module.

### 2.7. Target Gene Prediction of Differentially Expressed miRNAs

The AnnoLnc2 platform, developed by Peking University, can fully annotate the sequence and structure, expression and regulation, function and interaction, and evolution and genetic association of human LncRNA in real time. It is an upgraded version of the previous generation platform AnnoLnc [18]. The miRCancer database is a miRNA-tumor association database constructed based on literature text mining, and through PubMed text mining, the miRNA-tumor association data are regularly updated [19]. The miRWalk database is a cross-prediction database developed by the Medical Research Center of Mannheim Medical School of Heidelberg University that can predict target genes by miRNA and predict miRNA by target genes [20].

The miRNA that interacts with Linc00472 was obtained by AnnoLnc2. Since the expression of Linc00472 is decreased in renal clear cell carcinoma, the expression of miRNA that interacts with Linc00472 should increase as a ceRNA. Then, the miRNAs that have been studied in ccRCC were collected through the miRCancer database, and the miRNAs obtained in AnnoLnc2 were further filtered to obtain more reliable results. The filtered miRNAs were predicted in the miRWalk database for target genes, correlated with coexpressed differential genes in PPI, and screened out miRNAs and their target genes that interact with Linc00472 and constructed a regulatory network, which was visualized by Cytoscope3.8 software. In addition, the coexpressed differential genes and the selected miRNAs in each group of modules were analyzed separately, and a regulatory network was constructed, which was visualized by Cytoscope3.8 software to predict key target genes.

### 2.8. Statistical Analysis

The normal distribution test was performed on the expression difference between the cancer tissues of 22 patients with ccRCC and the paired adjacent normal tissues. If the normal distribution is met, the paired *t*-test is used for analysis; if the normal distribution is not met, then after correction the paired *t* test was used for analysis. According to the expression level of Linc00472 in cancer tissues, it was divided into the high-expression group and the low-expression group with the median as the cutoff point. Fisher's exact test was used to analyze the correlation between the expression of Linc00472 and clinicopathological indicators, including gender, age, tumor size, and pathological grade. When *P* < 0.05, it is considered statistically significant. The statistical software is GraphPad Prism 8.0 and IBM SPSS 25.

## 3. Results

### 3.1. Differentially Expressed LncRNAs and Protein-Coding Genes in ccRCC

Figure 1(a) is a volcano map of LncRNA differentially expressed in KIRC retrieved from the Cancer RNA-Seq Nexus database. The screening criterion is ∣log2 (Fold Change)∣ ≥ 1, and *P* < 0.01 after correction.  Figure 1(b) is a heat map of differentially expressed LncRNAs that meet the screening criteria in grade I to IV cancer tissues and adjacent tissues. A total of 359 differentially expressed LncRNAs that met the criteria were screened, of which 243 were upregulated and 116 were downregulated. A total of 1245 protein-coding genes that meet the criteria for differential expression were screened, of which 679 were upregulated and 566 were downregulated.

### 3.2. The Significantly Lower Expression of Linc00472 Is Associated with High Grade and Prognosis

We excluded LncRNAs that were not differentially expressed in grade I to IV cancer tissues. When the selected genes are closely related to the patient's prognosis, it will be more valuable for research. According to research of Wang et al. [15], 11 LncRNAs, 3 mRNAs, and 3 miRNAs in ccRCC are related to overall survival; 4 LncRNAs and 1 mRNA are verified as independent prognostic factors, of which Linc00472 is in ccRCC and was not studied in depth. Combined with our screening results, we noticed that the expression of Linc00472 in grade I to IV cancer tissues differed greatly, and its log2 (fold change) was −2.17, −2.25, −2.69, and −2.85. In order to observe the expression of Linc00472 more intuitively, the expression level of Linc00472 in 31 types of tumors and normal tissues was obtained through GEPIA2 analysis (Figure 2(a)), and it can be observed that the expression of Linc00472 in ccRCC is significantly reduced. As shown in Figure 2(b), analyzing the expression level of Linc00472 in 523 cancer tissues and 72 adjacent tissues, the expression of Linc00472 in cancer tissues was significantly reduced (*P* < 0.05). After analyzing the expression level of Linc00472 in cancer tissues of different pathological grades, it was found that the expression of Linc00472 was higher in grades I and II than in grades III and IV (Figure 2(c)).

We also analyzed the relationship between the expression level of Linc00472 and prognosis in GEPIA2. As shown in Figure 2(d) and Figure 2(e), the patients in the Linc00472 high-expression group must be in overall survival (OS) or disease-free survival (DFS). It is significantly better than the patients in the low-expression group. The expression level of Linc00472 is closely related to the prognosis of patients (*P* < 0.05), suggesting that Linc00472 may be an independent prognostic indicator of ccRCC.

### 3.3. Linc00472 Is Lowly Expressed in ccRCC Tissues and Associated with High Grade

In order to verify the analysis results of the TCGA database, we performed qRT-PCR verification on the cancerous tissues of 22 patients with ccRCC and their paired adjacent normal tissues (Figure 3). The pairing was performed after natural log correction.  Table 1 showed that the expression of Linc00472 was decreased in ccRCC tissues (*P* < 0.0001). We divided 22 patients into the high-expression group and the low-expression group according to the median expression level of cancer tissues of 22 patients. The statistical results show that the expression level of Linc00472 has no significant correlation with patient gender (*P*=1.000), age (*P*=0.387), and tumor size (*P*=0.395), and the expression level of Linc00472 in grade I and II cancer tissues was significantly higher than that in grade III and IV cancer tissues (*P*=0.024). This indicates that the expression level of Linc00472 is closely related to Furman nuclear grade of renal clear cell carcinoma, suggesting that Linc00472 plays an important role in the progression of ccRCC.

### 3.4. Enrichment Analysis of Linc00472 Coexpressed Differential Genes

LncRNA can regulate target genes through a variety of ways to exert its biological functions. In order to study the possible impact of Linc00472 coexpressed genes on the occurrence and development of ccRCC, we screened the protein-coding genes that were coexpressed with Linc00472 downloaded from the Co-LncRNA database, and performed GO BP and downregulated differentially coexpressed genes, respectively. The results of KEGG Pathway Enrichment Analysis showed that there were 998 coexpressed genes that were differentially expressed in grade I to IV cancer tissues and adjacent tissues, including 519 upregulated genes and 479 downregulated genes. The results of GO BP and KEGG Pathway enrichment analysis are shown in Figure 4. Among them, the GO BP analysis of the upregulated coexpressed differential gene showed that it is mainly involved in immune response, interferon-gamma-mediated signaling pathway, inflammatory response, angiogenesis, response to hypoxia, and other processes (Figure 4(a)). KEGG Pathway analysis results show that it is enriched in a variety of diseases and pathways, such as *Staphylococcus aureus* infection, viral myocarditis, allograft rejection, graft-versus-host disease, antigen processing and presentation, etc. (Figure 4(b)). The GO BP analysis results of the downregulated coexpressed differential genes showed that they are mainly involved in the metabolic process, fatty acid beta-oxidation, tricarboxylic acid cycle, oxidation-reduction process, gluconeogenesis, and other processes (Figure 4(c)). KEGG Pathway analysis results show that it is mainly enriched in metabolic pathways (Figure 4(d)). The enrichment analysis results of GO BP and KEGG Pathway suggest that differential genes coexpressed with Linc00472 may have an impact on the key process of tumorigenesis and development. An in-depth study of Linc00472 may provide favorable conditions for further revealing the molecular mechanism of renal clear cell carcinoma.

### 3.5. PPI Network Construction and Functional Module Analysis

In order to further understand the interaction between the differential genes coexpressed with Linc00472, and to find genes that may play a major function in the Linc00472 regulatory network, we used the STRING server to associate 998 coexpressed differential genes with Cytoscope3.8 software to perform visualization (Figure 5(a)). A total of 578 nodes and 2225 edges were obtained. Some of the nodes have a high degree of association, such as APP, degree = 53; GNAI1, degree = 30 in downregulated genes. However, most of the genes with a high degree of association are upregulated genes, such as C3, degree = 44; C3aR1, degree = 36; B2M, degree = 41; HLA-A, degree = 36, HLA-E, degree = 36; HLA-C, degree = 35; HLA-DRB1, degree = 35; and HLA-DRA, degree = 35. In addition, after MCODE analysis, the first two modules selected from the PPI network are shown in Figure 5(b). Module 1 has 40 nodes, 390 edges, and a function score of 20; Module 2 has 66 nodes, 481 edges, and a function score of 14. The GO BP and KEGG Pathway analysis results of the significantly enriched coexpressed genes in the two modules are shown in Table 2. In Module 1, most genes are clustered in immune response and interferon-gamma-mediated signaling pathway, accounting for more than 50%, while the results of KEGG have no obvious specificity. In Module 2, the results of GO and KEGG account for a small proportion.

### 3.6. Target Gene Prediction of miRNA Interacting with Linc00472

In order to further study the complete action path of Linc00472, it is also necessary to find miRNAs that interact with Linc00472 as a ceRNA. By predicting the target genes of miRNAs, the possible Linc00472-miRNA-mRNA pathways can be screened out of the differential genes coexpressed with Linc00472. The miRNAs that interact with Linc00472 we obtained in AnnoLnc2 were filtered by miRCancer database, and their target genes were predicted by miRWalk and correlated with coexpressed differential genes in the PPI network. A total of 42 miRNAs that interact with Linc00472 were obtained, and a network of miRNAs and their target genes was constructed (Figure 6(a)). In order to observe the key target genes more intuitively, we screened out miRNAs and their target genes in two modules (Figure 6(b)). Module 1 has 31 miRNAs interacting with Linc00472 and 26 target genes; Module 2 has 39 miRNAs interacting with Linc00472 and 53 target genes.

## 4. Discussion

There are few studies on Linc00472 in renal clear cell carcinoma, and there are still many blanks on what function it plays in ccRCC. Therefore, studying the mechanism of Linc00472 is of great significance in the diagnosis and treatment of ccRCC. Wang et al. [21] conducted a network analysis of ceRNA in ccRCC and found that 11 LncRNA, 3 mRNA, and 3 miRNA were related to overall survival; 4 LncRNA and 1 mRNA were verified as independent prognostic factors. It also contains Linc00472 of this research, and the result is consistent with the analysis result of this research. In this study, the expression level of Linc00472 in clinical samples was verified, and it was found that the expression level of Linc00472 was lower in higher grade cancer tissues, which was consistent with the results of data analysis in TCGA. For Linc00472 to become an independent prognostic factor in ccRCC, further observation and follow-up are needed to verify.

Linc00472 has also done some research in other tumors (lung cancer, colorectal cancer, liver cancer, breast cancer, etc.) [22]. Zou et al. [23] found that Linc00472 played a tumor suppressor effect in the KLLN-mediated p53 signaling pathway by downregulating the expression of miRNA-149-3p and miRNA-4270 in nonsmall cell lung cancer. Mao et al. [24] found that Linc00472 can inhibit the growth of lung cancer cells by downregulating the expression of miR-196b-5p. Su et al. [25] found that Linc00472 inhibited the proliferation of lung adenocarcinoma cells and promoted their apoptosis by downregulating the expression of miR-24-3p and DEDD (death effect domain protein). In colorectal cancer, Linc00472 may be downregulated due to hypermethylation of DNA [26], by downregulating the expression of miR-196a to upregulate the expression of PDCD4 (apoptosis-related protein 4), exerting a tumor suppressor effect [27]. Also in liver cancer, Linc00472 inhibits the proliferation, migration, and invasion of liver cancer cells through the miR-93-5p/PDCD4 pathway [28]. In breast cancer, the expression of Linc00472 is also regulated by promoter methylation [29], in which ER*α* (estrogen receptor *α*) can inhibit the phosphorylation of NF-*κ*B by upregulating the expression of Linc00472 [30]. In addition, Zhang et al. [31] found that the downregulation of Linc00472 can reduce the expression of FOXO1 through miR-300 and promote the occurrence of osteosarcoma.

LncRNA is a noncoding RNA with a length of more than 200 nucleotides. It has a wide range of biological functions and can affect a variety of signaling pathways, but not all of them are critical pathways. Therefore, we need to combine current research to find the most likely key pathways. For the above research, this study also found that Linc00472 interacts with miR-24-3p. According to reports, the expression level of miR-24-3p is elevated in a variety of malignant tumors, including lung cancer [32–34], liver cancer [35], breast cancer [36], bladder cancer [37], nasopharyngeal cancer [38] etc., is considered to be an oncogene. Therefore, it may also act as a ceRNA that interacts with Linc00472 to promote tumor cell proliferation, migration, and invasion in ccRCC. The main genes regulated by miR-24-3p in the two modules are HLA-DPB1, CXCL9, PLOD3, SLC2A5, STK10, TNFRSF1B, CD36, COL4A1, and SERPINA1. Among them, HLA-DPB1 and CXCL9 are the genes screened in Module 1, and the rest are the genes screened in Module 2 [39].

HLA-DPB1 is a member of HLA-II antigens, while HLA (human leukocyte antigen) is the human MHC (major histocompatibility complex). HLA is divided into three subclasses: class I antigens, including classical HLA-A, HLA-B, and HLA-C with high polymorphism, and nonclassical HLA-E, HLA-F, and HLA-G with limited polymorphism; Class II Antigens, including HLA-DPA1, HLA-DPB1, HLA-DQA1, HLA-DQA2, HLA-DQB1, HLA DQB2, HLA-DRA, HLA-DRB1, HLA-DRB2, HLA-DRB3, HLA-DRB4 and HLA-DRB5, as well as low variability involved in antigen processing and presentation Genes; Class III antigens, including genes related to inflammation, white blood cell maturation, and the complement cascade [40]. HLA is a presentation molecule of endogenous and exogenous antigens, and is widely involved in the process of human immune response. During the development of cancer, the immune system processes tumor cells through the three stages of immune editing (i.e, clearance, balance, and escape). In the end, tumors will escape the control of the immune system, leading to complete uncontrolled growth and widespread metastasis [41]. Tumor cells escape through a variety of mechanisms, including low expression of tumor surface antigens, making it difficult for the immune system to monitor them; the secretion of immunosuppressive factors (such as transforming growth factor beta, interleukin-10) and different regulation and induction of sexual lymphocytes or myeloid cells (such as regulatory T cells, bone marrow-derived suppressor cells); and downregulation or complete loss of HLA-I antigen expression to avoid the recognition and killing of cytotoxic T cells [42]. In this study, the expressions of HLA-I antigens screened from the PPI network were all upregulated, indicating that ccRCC cells may not completely trigger the immune escape mechanism through the downregulation or loss of HLA-I antigen expression. The carcinogenesis of cells is not only related to the change of HLA-I antigens but also related to the expression of HLA-II antigens. According to reports, more than 80% of breast ductal carcinomas lack the expression of HLA-II antigens [43]. In contrast, approximately 50% of papillary thyroid cancers and 60% of primary melanomas express HLA-II antigens, indicating increased expression of HLA-II antigens in these tumor types [44, 45]. The prognosis of different tumors is also related to the expression of HLA-II antigens. In colorectal cancer [46–48], laryngeal cancer [49], oropharyngeal cancer [50], HLA-II antigens are highly expressed and have a good prognosis. In melanoma and cervical cancer, HLA-II antigens are also highly expressed, but the prognosis is poor [51, 52]. The heterogeneity of HLA-II antigen expression in different tumors and the different prognosis indicate that it can play different roles in different tumors. In this study, the expression of HLA-II antigens in ccRCC is upregulated, indicating that it may play an important role in the development of ccRCC and affect the prognosis of patients. From the enrichment results of Module 1, it can be seen that, in the immune response, MHC class II antigen processing, peptide or polysaccharide antigen presentation, antigen processing and presentation, and other significant enrichment processes, HLA-II antigens are involved and play an important role in functional modules. Therefore, miR-24-3p may promote the progress of ccRCC by upregulating HLA-DPB1, which needs further verification.

CXCL9 is also known as interferon-*γ* (IFN-*γ*)-induced monocytes, which is a selective ligand of CXCR3 (CXC subfamily chemokine receptor 3), and CXC subfamily is one of the four subfamilies of chemokines (CC, CXC, CX3C, and XC). The CXCL9‐CXCR3 pathway can exert antitumor effects. In melanoma, the tumor area with high expression of CXCL9 has significant T-cell infiltration, which may be necessary to control tumor growth through IFN-*γ*-dependent pathways [53]. Another study found that CCL5 required for T cell infiltration was amplified by CXCL9 secreted by myeloid cells mediated by IFN-*γ*. Tumors that cohighly express CCL5 and CXCL9 show higher immune reactivity and a higher possibility of blocking immune checkpoints [54]. In skin tumors, lack of CXCL9 can still produce CXCL10, but cannot recruit cytotoxic CD8+ T cells, which leads to tumor generation and promotes tumor growth [55]. On the other hand, CXC chemokines that do not contain ELR (glutamate, leucine, and arginine) such as CXCL9 can inhibit angiogenesis. In nonsmall cell lung cancer cells, the overexpression of CXCL9 can inhibit tumor progression and metastasis by reducing tumor-derived blood vessel density [56]. It has also been confirmed in animal models that the combination of CXCL9 and low-dose cisplatin can inhibit angiogenesis and induce tumor cell apoptosis [57]. However, in humans, there are at least three mRNA splice variants of CXCR3, i.e., CXCR3A, CXCR3B, and CXCR3-alt. Among them, CXCR3A and CXCR3B combined with CXCL9 play a role in the regulation of angiogenesis. Overexpression of CXCR3B can promote the apoptosis of microvascular endothelial cells and inhibit angiogenesis. However, the overexpression of CXCR3A can enhance cell viability, promote proliferation, and enhance the ability of blood vessel formation [58]. This indicates that CXCL9-CXCR3 has a two-way regulatory effect on tumors and can promote tumor invasion and migration. Also in melanoma, CXCL9 can promote tumor migration through chemotaxis [59]. Adding exogenous CXCL9 to tongue squamous cell carcinoma cells expressing CXCR3 can promote cell invasion and migration as well as the EMT process [60]. In addition, it has been reported that prostate cancer cells recruit more CD4+ T cells by secreting more CXCL9. The recruitment of CD4+ T cells into the tumor may lead to increased invasion ability of prostate cancer cells [61]. Therefore, CXCL9 can not only play an antitumor effect but also promote tumor growth and metastasis, both of which can regulate tumor development. In this study, the expression of CXCL9 was upregulated, indicating that CXCL9 may have a relatively dominant role in promoting tumor growth and metastasis in ccRCC. From the enrichment results of Module 1, it can be seen that CXCL9 plays a role in the significantly enriched interferon-*γ*-mediated signal pathway and inflammatory response process, and may also be an important factor affecting the function of Module 1. Therefore, miR-24-3p may play the role of CXCL9 in promoting tumors by upregulating the expression of CXCL9, thereby promoting the growth and metastasis of ccRCC cells.

In Module 2, there are 7 genes regulated by miR-24-3p, which are PLOD3, SLC2A5, STK10, TNFRSF1B, CD36, COL4A1, and SERPINA1. The expression of PLOD3 (lysine hydroxylase 3) is increased in a variety of tumors, including lung cancer, liver cancer, and gastric cancer. In lung cancer, PLOD3 can promote the metastasis of lung cancer by regulating STAT3, and inhibiting the expression of PLOD3 can have an antitumor effect by regulating the PKC-*δ* signaling pathway [62, 63]. In liver cancer, PLOD3, BANF1, and SF3B4 are jointly selected as molecular markers for early diagnosis and screening of liver cancer [64]. In gastric cancer, the overexpression of PLOD3 is associated with the poor prognosis of gastric cancer [65]. The increased expression of PLOD3 in ccRCC suggests that it may play a role in the occurrence and development of ccRCC. SLC2A5 is the gene encoding fructose transporter 5 (GLUT5). Studies have shown that the high expression of GLUT5 in ccRCC aggravates tumor cell proliferation and colony formation [66]. TNFRSF1B is the coding gene of TNFR2 (Tumor Necrosis Factor Receptor II), and TNFR2 has been considered as a new target for tumor immunotherapy [67]. The immunotherapy targeting TNFR2 in ccRCC needs further research. CD36 is a fatty acid translocase, which plays an important role in the transport of long-chain fatty acids. The latest research found that CD36 is selectively upregulated in regulatory T cells in tumors. Knockout of CD36 reduced regulatory T cells enhanced the antitumor activity of lymphocytes infiltrated in the tumor, inhibited tumor growth, but did not destroy immune homeostasis [68]. In ccRCC, the high expression of CD36 has been verified, and it is positively correlated with visceral fat content, indicating a poor prognosis for patients [69]. CD36 may play an important role in the occurrence and development of ccRCC, and its influence on fat metabolism needs further study. COL4A1 (type IV collagen *α*1) can be used as a prognostic biomarker in urothelial carcinoma [70], According to the results of the ceRNA network analysis of ccRCC by Zheng et al. [15], COL4A1 is related to the overall survival of patients. Whether COL4A1 can be used as a prognostic marker for ccRCC needs further verification. SERPINA1 is a gene encoding AAT (*α*-1 antitrypsin), which is highly expressed in nonsmall cell lung cancer and plays an active role in the development of lung cancer [71]. Whether the high expression of SERPINA1 in ccRCC also plays a positive role in the development of ccRCC needs further verification. In short, the genes regulated by miR-24-3p in Module 2 are all upregulated genes, and the functional enrichment score is lower than that in Module 1. From the results of enrichment, only COL4A1 is significantly enriched in the catabolism of extracellular matrix and collagen. The development process of tumors is complex; these genes may also play a role in ccRCC through the regulation of miR-24-3p, and the main functions may be HLA-DPB1 and CXCL9. However, recent research on TNFR2 and CD36 has made new progress, and COL4A1 may also become a new prognostic marker. This has produced new ideas for studying the mechanism of ccRCC and is worthy of further study.

It can be observed from the PPI network that upregulated genes, except for the various subtypes of HLA, are C3, C3aR1, and B2M with the highest degree of association, which are all located in Module 1. According to the target gene prediction of Module 1, the only upregulated gene is C3aR1. Recent studies have shown that in purified vascular endothelial cells, the function of VEGFR2 requires the simultaneous presence of C3aR1/C5aR1 and IL-6R-gp130 signal transduction. And, in animal models, enhancing C3aR1/C5aR1 signal transduction will accelerate angiogenesis [72]. VEGFR2 can combine with VEGFA to regulate angiogenesis, and affect tumor growth and metastasis through the HIF pathway. Based on the results of target gene prediction, it is observed that C3aR1 and VEGFA are jointly regulated by miR-221-3p. The enrichment results of Module 2 also showed significant enrichment in angiogenesis and response to hypoxic conditions. Studies have explored the effect of high expression of miR-221-3p in ccRCC on the efficacy of TKI. Overexpression of miR-221-3p is associated with poor progression-free survival, while VEGFR2 is associated with longer survival [73, 74]. Then, whether miR-221-3p can be used as a ceRNA that interacts with Linc00472 in ccRCC to change the expression level of VEGFR2 by upregulating C3aR1, thereby regulating the growth and metastasis of ccRCC through the HIF pathway, needs further verification. APP and GNAI1 have the highest degree of association between downregulated genes, which are also located in Module 1. However, the enrichment results show that downregulated genes are significantly enriched in various metabolic processes, and APP and GNAI1 are not involved. Moreover, according to the analysis results, the genes that may play an important role in Module 1 are all upregulated genes, indicating that although APP and GNAI1 are highly correlated, they do not perform important functions. Therefore, we focused on the genes that are upregulated in the PPI network.

As mentioned in the previous article, HLA-II antigens may play an important role in the entire functional module, so we have paid attention to miR-17-5p. As shown by the target gene prediction results, miR-17-5p targets and regulates the expression of HLA-DQA1 and HLA-DQB1, as well as the expression of C3aR1 and C5aR1. Studies have found that the expression level of miR-17-5p in ccRCC is upregulated, its target is TRIM8, and it can connect p53 to the N-MYC pathway. Overexpression of miR-17-5p can inhibit TRIM8. On the one hand, it leads to a decrease in the stability of p53 tumor suppressor protein; on the other hand, it activates the oncogene N-MYC and promotes tumor cell proliferation [75]. In this study, miR-17-5p may affect the proliferation, migration, and invasion of ccRCC cells by upregulating the expression of HLA-DQA1 and HLA-DQB1; on the other hand, it may increase the expression of C3aR1 and C5aR1 in the classical HIF pathway. Linc00472 may also play an important role as a ceRNA that interacts with it.

In conclusion, the expression level of Linc00472 in ccRCC tissues is significantly lower than that in normal tissues adjacent to the cancer. Its low expression is related to Furman's high grade and poor prognosis. The results of protein interaction and functional enrichment analysis indicate that genes upregulated in ccRCC may play a major role. Analysis of target gene prediction results indicated that Linc00472 may act as ceRNA in miR-24-3p-HLA-DPB1 pathway, miR-24-3p-CXCL9 pathway, miR-221-3p-C3aR1-VEGFR2 pathway, miR-17-5p-HLA -DQA1/HLA-DQB1 pathway, and miR-17-5p-C3aR1/C5aR1-VEGFR2 pathway, and play an important role. In addition, the regulatory relationship between miR-24-3p and TNFR2, CD36 and COL4A1 should also be noted. In the next research, we will continue to expand the number of tissue samples to verify, and regularly follow-up, matched patients to analyze the prognosis, and verify the pathways that may play an important role at the cellular level and animal models, and closely integrate with the clinic to explore the role of Linc00472 in the diagnosis and treatment of ccRCC.

## Figures and Tables

**Figure 1:** Differentially expressed LncRNA in tumor tissues and adjacent normal tissues. (a) The volcano map of LncRNA differentially expressed in tumor tissues and adjacent normal tissues, the screening standard is ∣log2 (Fold Change)∣ ≥ 1, and *P* < 0.01 after correction. The blue dot on the left represents the downregulated LncRNA in cancer tissue, and the red dot on the right represents the upregulated LncRNA in cancer tissues. (b) The heat map of differential expression of LncRNA that meets the screening criteria in grade I to IV cancer tissues and adjacent tissues. Green represents downregulated LncRNA, and orange represents upregulated LncRNA. Red represents relatively high expression in tumor tissues and adjacent normal tissues, and blue represents relatively low expression. The greater the color difference, the more significant the difference in expression.

**Figure 2:** The expression level of Linc00472 in the TCGA database and its relationship with patient prognosis. (a) The expression level of Linc00472 in 31 tumor tissues and adjacent normal tissues. (b) The expression level of Linc00472 in 523 tumor tissues and 72 adjacent normal tissues. (c) The expression level of Linc00472 in grade I–IV cancer tissues. (d) The relationship between the expression level of Linc00472 and the overall survival of patients. (e) The relationship between the expression level of Linc00472 and the patient's disease-free survival.

**Figure 3:** The expression level of Linc00472 in ccRCC tissues is lower than that of matched adjacent normal tissues.

**Figure 4:** Analysis results of GO BP and KEGG Pathway coexpressed differential genes with Linc00472. (a) GO BP analysis results of upregulated coexpressed differential genes. (b) Upregulated coexpressed differential gene KEGG Pathway analysis results. (c) GO BP analysis results of downregulated coexpressed differential genes. (d) KEGG Pathway analysis results of downregulated coexpressed differential genes.

**Figure 5:** PPI network construction and module analysis. (a) PPI network. The node size represents the degree of interaction with other genes. The larger the node, the higher the degree of interaction. The red nodes represent upregulated genes, and the blue nodes represent downregulated genes. The depth of the node color represents the expression level of the gene, and the width of the edge represents the correlation score of the two genes, that is, the closeness of the correlation. (b) The first two modules selected by MCODE. Red represents upregulated genes, and blue represents downregulated genes. The shade of the node color represents the expression level of the gene, and the width of the edge represents the correlation score of the two genes.

**Figure 6:** miRNA interacts with target genes in a network. Pink represents miRNAs that interact with Linc00472, red represents upregulated target genes, and blue represents downregulated target genes. (a) Interaction network of all miRNAs and target genes. (b) miRNA and target gene interaction network in two modules.

**Table 1:** The correlation between the expression level of Linc00472 and the clinicopathological characteristics of patients.

Clinicopathological characteristics	Total (*n* = 22)	Linc00472 expression level		*P*
		Low	High	
Gender				1.000
Male	16	8 (50%)	8 (50%)	
Female	6	3 (50%)	3 (50%)	

Age				0.387
<55	9	6 (66.7%)	3 (33.3%)	
≥55	13	5 (38.5%)	8 (61.5%)	

Tumor size (cm)				0.395
<5	11	4 (36.4%)	7 (63.6%)	
≥5	11	7 (63.6%)	4 (36.4%)	

Furman classification				0.024^∗^
I, II	14	4 (28.6%)	10 (71.4%)	
III, IV	8	7 (87.5%)	1 (12.5%)	

^*∗*^ *p* < 0.05.

**Table 2:** Significantly enriched GO BP and KEGG Pathway analysis results in the two modules.

Module		Description	*P*. adjust	Counts
Module 1	GO BP terms	Immune response	1.08947*E* − 17	24
		Interferon-gamma-mediated signaling pathway	3.01473*E* − 15	21
		Inflammatory response	1.71115*E* − 12	10
		Antigen processing and presentation of peptide or polysaccharide antigen via MHC class II	1.80454*E* − 10	8
		Antigen processing and presentation	2.03552*E* − 10	12
		Type I interferon signaling pathway	1.77292*E* − 08	8
	KEGG Pathway	*Staphylococcus aureus* infection	1.0228*E* − 20	14
		Viral myocarditis	5.11466*E* − 15	14
		Allograft rejection	6.1499*E* − 14	13
		Graft-versus-host disease	1.54791*E* − 13	13
		Antigen processing and presentation	2.32687*E* − 13	15
		Phagosome	5.89325*E* − 12	14
		Type I diabetes mellitus	1.08722*E* − 11	13
		Autoimmune thyroid disease	2.98279*E* − 11	13

Module 2	GO BP terms	Angiogenesis	7.80442*E* − 13	7
		Extracellular matrix organization	6.35682*E* − 12	16
		Response to hypoxia	1.17332*E* − 11	5
		Type I interferon signaling pathway	1.77292*E* − 08	6
		Platelet degranulation	2.34138*E* − 08	14
		Collagen catabolic process	1.60661*E* − 07	11
		Defense response to virus	1.66166*E* − 07	5
	KEGG Pathway	Focal adhesion	1.64514*E* − 07	13
		ECM-receptor interaction	3.56477*E* − 06	12

Immune response*:* CXCL10, B2M, APLN, C5AR1, HLA-A, HLA-C, HLA-B, HLA-E, HLA-DQA2, HLA-DQA1, HLA-F, HLA-DPA1, GBP2, HLA-DRA, HLA-DQB1, GPR183, HLA-DRB1, C3; interferon-gamma-mediated signaling pathway: HLA-DQB1, ICAM1, HLA-DRB1, HLA-A, IFI30, HLA-C, OAS1, HLA-B, OAS2, HLA-E, HLA-DQA2, HLA-DQA1, HLA-F, B2M, CD44, HLA-DRB5, HLA-DPA1, HLA-DPB1, GBP2, GBP1, HLA-DRA, CXCL9, OAS1, OAS2; inflammatory response: C3AR1, C3, FPR1, CXCL9, FPR3, CXCL10, CCL20, CXCR4, C5AR1, ANXA1; antigen processing and presentation of peptide or polysaccharide antigen via MHC class II: HLA-DQB1, HLA-DRB1, HLA-DRB5, HLA-DPA1, HLA-DPB1, HLA-DQA2, HLA-DQA1, HLA-DRA; antigen processing and presentation: HLA-DQB1, HLA-DRB1, HLA-A, HLA-C, HLA-B, HLA-E, HLA-DQA2, HLA-DQA1, HLA-DRB5, HLA-DPA1, HLA-DPB1, HLA-DRA; type I interferon signaling pathway: HLA-A, HLA-C, OAS1, HLA-B, OAS2, HLA-E, HLA-F, GBP2; *Staphylococcus aureus* infection: HLA-DQB1, C3AR1, HLA-DRB1, C3, FPR1, FPR3, HLA-DRB5, HLA-DPB1, ICAM1, C5AR1, HLA-DQA2, HLA-DQA1, HLA-DPA1, HLA-DRA; viral myocarditis: HLA-DQB1, ICAM1, HLA-DRB1, HLA-A, HLA-C, HLA-B, HLA-E, HLA-DQA2, HLA-DQA1, HLA-F, HLA-DRB5, HLA-DPA1, HLA-DPB1, HLA-DRA; allograft rejection: HLA-DQB1, HLA-DRB1, HLA-A, HLA-C, HLA-B, HLA-E, HLA-DQA2, HLA-DQA1, HLA-F, HLA-DRB5, HLA-DPA1, HLA-DPB1, HLA-DRA; graft-versus-host disease: HLA-DQB1, HLA-DRB1, HLA-A, HLA-C, HLA-B, HLA-E, HLA-DQA2, HLA-DQA1, HLA-F, HLA-DRB5, HLA-DPA1, HLA-DPB1, HLA-DRA; antigen processing and presentation: HLA-DQB1, HLA-DRB1, HLA-A, IFI30, HLA-C, HLA-B, HLA-E, HLA-DQA2, HLA-DQA1, HLA-F, B2M, HLA-DRB5, HLA-DPA1, HLA-DPB1, HLA-DRA; phagosome: HLA-DQB1, HLA-DRB1, C3, HLA-DRB5, HLA-DPB1, HLA-A, HLA-C, HLA-B, HLA-E, HLA-DQA2, HLA-DQA1, HLA-F, HLA-DPA1, HLA-DRA; type I diabetes mellitus: HLA-DQB1, HLA-DRB1, HLA-A, HLA-C, HLA-B, HLA-E, HLA-DQA2, HLA-DQA1, HLA-F, HLA-DRB5, HLA-DPA1, HLA-DPB1, HLA-DRA; autoimmune thyroid disease: HLA-DQB1, HLA-DRB1, HLA-A, HLA-C, HLA-B, HLA-E, HLA-DQA2, HLA-DQA1, HLA-F, HLA-DRB5, HLA-DPA1, HLA-DPB1, HLA-DRA; angiogenesis: SERPINE1, COL8A1, FN1, COL4A2, COL15A1, VEGFB, VEGFA; extracellular matrix organization: ITGB2, COL6A3, SERPINE1, COL6A2, COL6A1, COL8A1, FN1, COL4A2, COL4A1, SPARC, COL5A2, COL5A1, VWF, COL1A2, VCAN, COL1A1; *Response to hypoxia*: TGFB1, PLOD1, PLOD2, VEGFB, VEGFA; type I interferon signaling pathway: BST2, SAMHD1, PSMB8, STAT2, ISG20, ISG15; platelet degranulation: ALDOA, CLU, SERPING1, SPARC, TGFB1, TIMP1, VEGFB, VWF, CD36, SERPINE1, VEGFA, SERPINA1, CFD, FN1; collagen catabolic process: COL4A2, COL4A1, COL6A3, COL1A2, COL6A2, COL15A1, COL6A1, COL1A1, COL8A1, COL5A2, COL5A1; defense response to virus: BST2, SAMHD1, STAT2, ISG20, ISG15; focal adhesion: COL6A3, COL6A2, COL6A1, FN1, COL4A2, COL4A1, COL5A2, COL5A1, VEGFB, VWF, VEGFA, COL1A2, COL1A1; ECM-receptor interaction: VWF, COL4A2, COL4A1, CD36, COL6A3, COL1A2, COL6A2, COL6A1, COL1A1, COL5A2, COL5A1, FN1.

## Data Availability

The data that support the findings of this study are available from the corresponding author upon reasonable request.
